This article has been retracted.

# Systematic Risk Analysis of Semiconductor Global Market Based on Deep Feature Fusion K-Means Algorithm

**DOI:** 10.1155/2022/8036956

**Published:** 2022-09-29

**Authors:** Wenjie Qiu

**Affiliations:** Graduate School, Keimyung University, Deagu 42601, Republic of Korea

## Abstract

As the global semiconductor industry has entered a new round of rapid growth, it has also entered a golden cycle of economic growth. Semiconductor companies increase their intrinsic value through financing, industry mergers and acquisitions, and venture capital searches. At the same time, market investors pay more attention to the intrinsic value of companies when looking for good investment targets. Therefore, the systematic risk assessment of the global semiconductor market has become a common concern of market investors and corporate management. In this context, this paper found a method that can assess the systemic risk of the semiconductor global market, which is to use the K-means algorithm based on deep feature fusion. This paper analyzed the algorithm in depth, analyzed the quantum space of tensors, and used the definition of cluster fusion to obtain the relationship between the projection matrices *U* and *V*. Experiments were carried out on the improved algorithm, and market research was conducted on a multinational semiconductor company A, which mainly included the basic statistics of the rate of return and the ACF and PACF coefficients of the rate of return series. Finally, the stock risk comparison of company A and company B in the same period was carried out. The experimental results showed that comparing the three items of compound growth rate, coefficient of variation, and active rate coefficient, the highest compound growth rate was 0.41, which came from Category 2, the highest variation coefficient was 2.31, which came from Category 10, and the highest active rate coefficient was 1.78, which came from Category 9. The experimental content was completed well.

## 1. Introduction

In the past two decades, China's semiconductor industry has developed rapidly, which is inseparable from the Chinese government's policy support for the semiconductor industry; the implementation of tax reduction policies has provided many tax incentives for foreign-invested semiconductor companies. The database can perform statistics, query, and input functions on data and even the future development trend of data. The driving force of market development still mainly comes from mobile phones, LCD TVs, and other electronic products with large output, and the market growth rate is expected to be around 20%. As China has become the world's electronic product manufacturing plant, there is a huge demand for semiconductor products. In recent years, major international semiconductor manufacturers have invested heavily in China, making China's market one of the most competitive markets. Of course, China's market is very important in the market strategies of international manufacturers. In the face of such a sudden change in the global semiconductor market, for every practitioner, this is an era of opportunities and risks. In addition to that, how to reasonably avoid risks and create value has become a hot topic in the industry. The ratio of the number of relevant correct retrieval images in the query result to the total number of all relevant retrieval images is called the recall rate, which has the characteristics of comprehensive retrieval. The images are classified, the associated images of each image in the image are judged, and the category of each image is used as the benchmark to measure the retrieval accuracy.

Zhang et al. proposed a CoES model based on the mean value of tail loss in the assessment of systemic risk in the semiconductor global market. This method focused more on the average of tail losses rather than the expected losses on individual quantiles compared with the traditional Co-VaR model; it can provide more accurate information for regulation when capturing systemic risks in the financial system [1]. Chiu et al. mainly discussed the Malmquist productivity index of Taiwan's semiconductor industry based on the meta-frontier method from the perspective of performance evaluation. From the perspective of dynamic productivity performance, they found that the main reason for the negative growth of IC packaging and testing companies and IC design companies was the backwardness of technological change, and the main reason for the negative growth of IC packaging and testing companies and IC design companies was the backwardness of technological change [2]. Betelin discussed the challenges and risks of forming a digital economy in Russia. The results showed that this was due to the lack of companies in the country that have the economic and social conditions to become global market leaders in semiconductors and radio electronics. Half of the global semiconductor market was controlled by U.S. companies that form the basis of the already formed “U.S. semiconductor digital economy,” of which Russia is a consumer [3]. In order to have a meaningful discussion on the future trends of electronic testing, Ooi tried to understand the trends of the semiconductor industry over the past two decades. The global semiconductor market saw tremendous growth from the early 1980s to the late 1990s, with an overall compound annual growth rate of 14.9%. During this period, the growing demand for integrated circuits pushed up prices and resulted in a large number of companies competing in the semiconductor market [4]. The research route of these experts and scholars is relatively traditional, the way of collecting data is not intelligent enough, and the designed system is often unable to meet the needs of a large amount of data impact. So, if there is a way to solve the above problem is a concern now. In view of the abovementioned important and difficult problems in the risk assessment of the semiconductor industry, this paper proposed to use the K-means algorithm to construct the system. Shen et al. proposed a feature plant image stitching method based on the color and depth information of the Kinect sensor. The effective plant parts in color images were extracted by using the K-means algorithm and plant depth information. Since the SURF algorithm is three times faster than the SIFT (scale invariant feature transform) algorithm, the SURF (accelerated robust feature) algorithm was used to extract the effective part [5]. Fan et al. proposed an improved sonar target detection and classification algorithm based on YOLOv4. First, the feature extraction network CSPDarknet-53 in YOLOv4 was improved to reduce model parameters and network depth. Second, the PANet feature enhancement module in the YOLOv4 model was replaced with an adaptive spatial feature fusion module (ASFF) to obtain better feature fusion effects [6]. Chen et al. introduced a new method called “K-Means Clustering-Driven N-Two-Stage Algorithmic Aggregation Paradigm” (N2S-KMC) to overcome the limitation of information distortion by reducing the cardinality in the first stage of the aggregation process. He believed that aggregating the HFLTS likelihood distribution under the framework of statistical data analysis can effectively reduce information loss and distortion [7]. Chen used the idea of K-means clustering to analyze the collected raw error data, such as the teacher level, teaching facility investment, and the policy relevance level. The data that the algorithm considers unreliable were removed, the remaining valid data were used to calculate the weight factor of the modified fuzzy logic algorithm, and the weighted average was evaluated by using the node measurement data; then, the final fusion value was obtained [8].

In response to this problem, this paper studied and established the default index model of individual customers through data mining and defined the basic elements of the model. A system was produced by using the K-means method; it has the ability to monitor the development of customers that may lead to the risk of due loan in advance and reduce the ability to repay the personal loan reserve. In addition to that, it can predict personal loan risks and effectively predict and control nonperforming balance sheet loan retail personnel and nonperforming loan ratios.

## 2. The Method of Deep Feature Fusion for Market Risk

### 2.1. Marketing

There are two advantages of sparsification: one is that it can automatically select features and another is that it has better interpretability, which is convenient for data visualization to reduce the amount of calculation and transmission and storage. Marketing is an organizational function and process capable of creating, disseminating, and delivering value to customers and managing customer relationships for the benefit of both the organization and its stakeholders [9]. It is also an administrative and social process in which collectives and individuals respond to their own wishes and needs by creating and exchanging products and values with others [10]. Marketing strategy is a process in which a company takes customer needs as its starting point, receives customer needs and purchasing power information based on relevant experience, and systematically organizes the company's various business activities and customer expectations. The satisfactory services and goods were provided to customers through coordinated pricing strategies, promotion strategies, product strategies, and channel strategies [11]. Under the macroeconomic background of the current global economy, the marketing theory has been continuously improved and developed with the changes of the market economy [12].

Whether it is a company or a specific business, decision makers must formulate strategies to guide its survival and development and must achieve a dynamic balance between organizational goals, internal conditions, and external environments [13]. Companies cannot address the threats and opportunities of the external environment alone. It must combine its own business objectives and internal conditions to identify appropriate opportunities for the company [14]. Opportunities in the environment can only be opportunities for a company if they are aligned with the resources and core competencies that belong or will belong to the company. If the good opportunities in the external environment do not match the company's capabilities and resources, the company should prioritize improving internal conditions [15]. The SWOT matrix is shown in Figure 1.

### 2.2. The Feature Algorithm for Deep Feature Fusion

The traditional method extracts the single image retrieval feature manually, where the single feature contains insufficient information and the retrieval result is poor. With the maturity of technical theory, multifeature fusion gradually replaces single feature, but its method still relies on manual feature extraction. The dynamic recognition framework based on depth map was introduced, which can simultaneously capture the shape and spatiotemporal characteristics of dynamic sequences and use this divergence to analyze systemic risks [16]. For this purpose, currently proposed low-level depth features are analyzed, while fusing relatively well-performing shape and spatiotemporal features [17]. For shape features, an important point is that the 3D structural information of the depth map should be fully utilized. The depth motion maps were used in the scheme to capture 3D structure and shape information based on this initial motivation [18]. Another important point is that because the dynamic characteristics are very fine, the shape information of the depth motion map must be enhanced to obtain the spatial-temporal-frequency variation [19]. In the scheme, the texture information and edge information of three depth motion maps were obtained through the DLE descriptor. DLE integrated the LBP and EOH features based on the depth motion map, which can effectively describe the texture and edge information of system risks in dynamic changes [20]. However, deep motion maps have some drawbacks. Due to the accumulation of the absolute difference of the projection maps of adjacent frames, the motion of the same spatial position will be overwritten. Another disadvantage is that deep motion maps cannot capture the before-and-after sequence of motion over time. The feature map of the convolutional layer uses the convolution kernel to convolve the feature map of the upper layer and obtains the output two-dimensional plane through a nonlinear function. The convolved values of several feature maps are combined into one output feature map. In the whole process, each layer involves the rate of change of the error to the basis, which is called the sensitivity, that is, the derivative.

In this case, spatiotemporal information is particularly important to improve the recognition rate. All the above problems can be solved by fusing spatiotemporal features. For spatiotemporal features, HOG2 has been verified in the field of gesture recognition and performs relatively well. In particular, its idea is very simple. In this fusion scheme, HOG2 was used to supplement the loss of temporal information in the depth motion map generation process and capture the detailed changes of information in the spatial and temporal domains, as shown in Figure 2.

The process is as follows: firstly, the depth motion map is extracted, the LBP histogram feature and EOH feature of the depth motion map are calculated, the shape information of the depth motion map is enhanced, its texture and edge information is obtained, and the DLE feature is obtained. Then, the spatiotemporal feature HOG2 is fused to obtain an effective descriptor, which is defined as the DLEH2 descriptor.

### 2.3. Tensor Subspace

Object retrieval, as one of the most important branches in the field of computer vision, aims to retrieve objects from image information quickly and accurately. It is also important for our systems to identify risks. A tensor is similar to a high-dimensional data model, which is an abstract physical quantity. It has obvious advantages in maintaining complex spatial structures, and it has been paid more and more attention by people. The tone can be seen as an extension of the table. The vector is the primary tone and the table is the secondary tone. Stacking several panels of the same size together to form a series of cubes is the tertiary tone. Higher-order tones cannot be directly described. High pressure analysis requires some functionality. Definitions of the relevant upper-class tone are given as follows:

Satisfaction:

(1) $$\begin{array}{c} \left\{\begin{array}{c} C_{i}\cap C_{j}=\emptyset ,i\neq j,\\ C_{1}\cup C_{2}\cup \ldots \cup C_{k}=X. \end{array}\right. \end{array}$$

The main functions for calculating distance are as follows:

(1) MinKowshi distance:
  (2) $$\begin{array}{c} d\left(x,y\right)={\left[\overset{k}{\underset{i=1}{\sum }}{\left(x_{i}-y_{i}\right)}^{t}\right]}^{1/t},t>0\text{.} \end{array}$$
(2) Horse distance:
  (3) $$\begin{array}{c} d\left(x,y\right)=\left(x-y\right)\sum i{\left(x-y\right)}^{\prime }\text{.} \end{array}$$
(3) Lance and Williams distance:
  (4) $$\begin{array}{c} d\left(x,y\right)=\overset{k}{\underset{i=1}{\sum }}\frac{\left|x_{i}-y_{i}\right|}{\left|x_{i}+y_{i}\right|}\text{.} \end{array}$$

The definition of cluster fusion is shown in Figure 3.

Pixels in an image were marked in decimal form, and the resulting image was called an LBP-encoded image. Finally, the histogram features of LBP-encoded images were computed to obtain texture information concisely.

In the fusion function,

(5) $$\begin{array}{c} S_{ij}=\frac{count\left(x_{i}\in \pi_{i}\in x_{j}\in \pi_{j}\right)}{k}\text{.} \end{array}$$

The coefficient of variation is calculated as follows:

(6) $$\begin{array}{c} CV=\frac{\sigma }{\bar{X}}\times 100\%\text{.} \end{array}$$

The ratio of the coefficient of variation to the correlation coefficient is expressed as follows:

(7) $$\begin{array}{c} g_{j}=\frac{1}{k-1}\overset{k-1}{\underset{i=1}{\sum }}\frac{CV}{\gamma_{ij}}\text{.} \end{array}$$

The index that is usually used to measure similarity is distance, and the measure that is commonly used in classification to measure the quality of classification is as follows:

(8) $$\begin{array}{c} {VRC}_{k}=\frac{SSB}{SSW}\times \frac{\left(N-k\right)}{\left(k-1\right)}\text{.} \end{array}$$

The optimal projection subspace is determined according to the eigenvector composition corresponding to the nonzero eigenvalues of the covariance matrix C. BI is expressed as follows:

(9) $$\begin{array}{c} BI=\frac{\sigma_{DAU}}{{\bar{X}}_{DAU}}\text{.} \end{array}$$

In recent years, the development of tensor PCA has solved the problems existing in the traditional PCA algorithm, improved the recognition accuracy, and has been widely used in image data processing. An image itself can be represented by a matrix or a two-dimensional tensor. The grading method uses the ratio of the average size of the industry to measure the importance of the industry as follows:

(10) $$\begin{array}{c} l_{i}=\frac{Y_{i}}{\overset{k}{\underset{i=1}{\sum }}Y_{i}}\text{.} \end{array}$$

The CNN is a network model composed of multiple hidden layers, where each hidden layer contains multiple planes, multiple planes represent a feature, respectively, and one plane contains multiple neurons and is independent of each other. After data transformation, the standardized expression of data transformation is shown as follows:

(11) $$\begin{array}{c} \hat{Y_{i}}=\frac{Y_{i}-\hat{Y}}{\sigma }\text{.} \end{array}$$

Then, the tensor product of *X* and *Y* is defined as follows:

(12) $$\begin{array}{c} {\left(x⊗y\right)}_{n_{1}\times n_{2}\times \ldots n_{m}\times n_{1}{}^{\prime }\times n_{2}{}^{\prime }\times \ldots n_{m}{}^{\prime }}=x_{n_{1}\times n_{2}\times \ldots n_{M}}y_{n_{1}{}^{\prime }\times n_{2}{}^{\prime }\times \ldots n_{M}{}^{\prime }}. \end{array}$$

The modulo *d* multiplication of a tensor is as follows:

(13) $$\begin{array}{c} {\left(x\times U^{d}\right)}_{i_{1\times }i_{2\times \ldots \times j\times i_{d+1}\times \ldots \times i_{M}}}=\underset{i\;d}{\sum }\left(x_{i_{1\times }i_{2\times \ldots \times j\times i_{d+1}}U_{j\times i_{d}}}\right)\text{.} \end{array}$$

*X* is represented in terms of two orthonormal bases as follows:

(14) $$\begin{array}{c} X=\underset{ij}{\sum }\left(u_{i}^{T}xv_{j}^{T}\right)u_{i}v_{j}^{T}\text{.} \end{array}$$

First, specifically, the image was filtered to remove noise. Secondly, widely used filters, such as Gaussian filter and median filter, were used to remove noise, and then, the edge detection algorithm was used to detect 4 oriented edges in the image. Finally, the relationship between the projection matrices *U* and *V* could be obtained as shown in the following formula:

(15) $$\begin{array}{c} \left(U^{*},V^{*}\right)=arg\begin{array}{c} \min\\ U,V \end{array}U\times Y\times V^{T}-X_{F}^{2}\text{.} \end{array}$$

After calculating the depth motion map, the LBP histogram feature and EOH feature of the depth motion map were extracted, which enhanced the shape information of the depth motion map and obtained rich shape cues including local texture and edge information of the depth motion map, which improved the discernment of the descriptor.

### 2.4. The Semiconductor Manufacturing Process Flow

Since the size of the integrated circuit chip components is in the nanometer scale, the control of contamination is extremely strict, so the entire production environment was located in a highly clean room with constant temperature and humidity. Integrated circuit manufacturing is the execution of a series of complex chemical or physical operations on a silicon wafer. Briefly, these operations can be divided into four basic categories: thin film fabrication (layer), patterning (pattern), etching, and doping. The wafer fabrication was finally completed by repeatedly repeating these four categories of operations.

In a wafer fab, it is generally subdivided into 6 separate production areas: diffusion (including oxidation, film deposition, and doping processes), lithography, etching, thin film, ion implantation, and polishing, as shown in Figure 4.

Semiconductor manufacturers need to have good production management strategies and plans to improve wafer fabrication processes and operations. Therefore, the research and optimization of this link are of great significance for wafer manufacturers to shorten the production cycle, improve production efficiency, and save costs, so as to win the market and gain profits in the fierce market competition.

## 3. Experiments on Systemic Risk in the Semiconductor Global Market

In 2021, when the global economy had turned into a cold winter with the arrival of the new crown epidemic, the total revenue of the semiconductor industry had ushered in a new peak. Total semiconductor industry revenue in 2021 was $586.8 billion, being $100 billion higher than the second-highest 2018 on record ($484.7 billion). Semiconductor industry revenue grew 24.2% year-over-year in 2021, the second-highest record since Omdia started tracking the metric in 2002. Under such circumstances, the detection of systemic risks in the global semiconductor market is particularly important.

### 3.1. Market Research

The market research was conducted on a multinational semiconductor company A, and the results are shown in Figure 5.

As shown in Figure 5, the mean of returns was very small, almost close to zero, and the difference between the median and the mean was large, which indicated that the distribution of returns is biased. The calculated skewness (Skewness) was 5.1795, which is greater than zero; it indicated that the return series is skewed to the right relative to the normal distribution. The results were retrieved from the dataset, as shown in Table 1.

It can be seen that when the feature dimension increased, the expected value was basically at a relatively high level. When the peak was 512, the expected value was 92.0. The ACF and PACF coefficients of the yield series were arranged, as shown in Figure 6.

It can be seen that in the lags 1 to 12, each period was not significant, and there was no significant correlation, and all ACF values were not significant at the 5% significance level.

### 3.2. Short-Term Impact of the Introduction of Stock Index Options on the Systemic Risk of the Global Semiconductor Market

The stock risks of Company A mentioned above with Company B in the same period were compared, *δ* is used as a measurement index, and the three months before, after three months, and six months of stock index options listing are used as the window period; 1 represents the first three months, 2 represents the last three months, and 3 represents the last six months, as shown in Figure 7.

Before the stock index option was launched, the mean value of the sample's systematic risk index *δ* was 0.1885512, and three months and six months after the stock index option was launched, the mean values of the sample's systematic risk index *δ* were 0.295638699 and 0.23656518, respectively, with an increase of 56.8% and 25.5%, respectively. It can be seen intuitively that after the introduction of stock index options, the proportion of systematic risk in stock risk has increased, that is, the systematic risk of stock market has also increased.

### 3.3. The System Performance Test of the K-Means Algorithm Based on Deep Feature Fusion

The correlation analysis function in R software was used to carry out correlation analysis on the selected data variables. The analysis results are shown in Table 2.

As shown in Table 2, the average scale and average MAU, average number of starts, and average usage time, the correlation coefficient reached more than 0.93; the correlation between the coefficient of variation and the coefficient of variation of times and time was as high as 87%; the retention rate and the unloading conversion rate were completely negatively correlated. Due to the large amount of data, the Nbclust package in R was used to analyze the number of classified clusters. The analysis diagram is shown in Figure 8.

The clustered App data was input, the number of clusters *k* = 11, and then the corresponding category and cluster center vector of each data was output. The results of data clustering are shown in Table 3.

As shown in Table 3, comparing the three items of compound growth rate, coefficient of variation, and active rate coefficient, the highest compound growth rate was 0.41, which came from Category2, the highest variation coefficient was 2.31, which came from Category10, and the highest active rate coefficient was 1.78, which came from Category9. The recommended number of clusters for the 26 indicators is shown in Figure 9 after using the K-means weighted clustering model.

It is divided into 9 categories using the K-means weighted clustering algorithm, and the results are shown in Table 4.

Then, we mark the center points of the weighted cluster centers in Table 4, as shown in Table 5.

As can be seen from Tables 4 and 5, the average size of Category 3, Category 4, Category 6, and Category 7 was smaller; among them, Category 7 had a faster growth rate, Category 3 and Category 6 were relatively stable, and Category 4 was shrinking. The average size of Category 1, Category 2, Category 5, and Category 9 was medium, of which Category 1 had a faster growth rate, Category 2 and Category 5 fluctuated slightly, and Category 9 was relatively stable. Category 8 had the largest average size and was the leading company in the semiconductor industry.

## 4. K-Means Method Application

### 4.1. The Text Clustering Module

The text clustering module was mainly used to implement clustering analysis on the text vectors that have completed text preprocessing. The text clustering module mainly includes two clustering methods, namely, K-means text clustering and Canopy-K-Means text clustering. While performing text clustering analysis, users need to configure corresponding parameters according to different algorithms to run the clustering analysis of the algorithm. In particular, the selection of parameters and other important factors affect the effect of retrieval. In the process of network training, good parameters that match the model are found to achieve a two-way balance between speed and accuracy in target retrieval, thereby improving the comprehensive performance of the model. These are all yet to be studied.

The K-means parameter configuration use case is similar to the Canopy-K-Means parameter configuration use case business process, except that K-means needs to configure the number of clusters K and the convergence threshold of the iterative process, while Canopy-K-Means needs to configure the division threshold T1 of the initial center selection and the convergence threshold of the iterative process.

If the word segmentation method based on statistics and machine learning is used, manual annotation needs to be performed before the text segmentation. When the amount of data is large, this method requires a lot of labor costs and does not meet the actual needs. The method based on mechanical word segmentation is fast and easy to implement, which is beneficial to improve the word segmentation efficiency of large-scale text data. Therefore, this paper adopted the method of mechanical word segmentation to segment the text data. Among them, IKAnalyzer has a faster word segmentation speed, which can process 600,000 Chinese characters per second, and its structure is relatively simple, users can add and formulate dictionaries according to actual needs. The accuracy rate of the IKAnalyzer tokenizer is also high. The current test data statistics can achieve an accuracy rate of 95%. It does not need to invest a lot of manpower for training and labeling, and it can customize the dictionary to facilitate the addition of words in specific fields. Therefore, IKAnalyzer was finally used to segment the text data.

### 4.2. Multiview Clustering Technology

Multikernel learning algorithms apply kernel functions to different physical angles and improve learning performance by combining linear or nonlinear kernel functions. The application of the subspace learning algorithm assumes that the portal perspective is created from a possible subspace, thereby obtaining a latent subspace shared by multiple perspectives. Since acquiring multiperspectives is the foundation of multiperspective learning, in addition to studying multiperspective learning models, ways to create and evaluate multiple perspectives are also very valuable. In general, learning from multiple perspectives has advantages over learning from a single perspective by exploring the consensus and mutuality of different perspectives.

Existing multiview clustering techniques are also divided into three following categories based on multiview learning methods compared with single-view clustering algorithms: standard collaborative training clustering algorithms, multicore learning clustering algorithms, and subspace learning clustering algorithms. Although there are significant differences between different approaches that combine multiple perspectives to improve learning performance, what they all have in common is the use of consensus or complementarity criteria to ensure that multiperspective learning can be successful. Therefore, combining these two criteria, considering not only the information of a single perspective, but also the complementary information that depends on each other, can achieve the purpose of making the clustering results more accurate.

### 4.3. Improvement of Initial Cluster Center Selection

The K-means clustering algorithm is the most commonly used clustering algorithm in data mining technology, and its division method is simple and efficient. When solving the clustering problem, typical sample points can be selected as the initial clustering centers of the clustering algorithm, so the selected clustering centers can be effectively prevented from being isolated points or edge noise points, and the possible disturbance problem of the clustering results can be solved, which can make the clustering result more accurate. The data objects from the dense area of the data set were selected as the initial cluster center, and the determination methods include selecting the cluster center, relying on experience selection, using density algorithm selection and so on. No matter which method was used to obtain the initial cluster center, the principle is to select the stable cluster with strong objectivity. The gradient method to find extreme values all search in the direction of decreasing energy. The division results should reflect the correlation between different data objects in the data set and also reflect the distribution characteristics between different data sets. The clustering algorithm is a kind of clustering analysis method based on objective function. Usually, the gradient method is used to obtain the minimum value of the function. Therefore, when choosing unreasonable initial cluster centers, it is easy to obtain local minimum value.

For the traditional K-means clustering algorithm, the selection of the initial cluster center directly affects the clustering results. Cluster analysis of data sets with large differences in shape is achieved through squared error and criterion functions. The most convenient way is to arbitrarily select multiple different initial values to run the algorithm, in order to reduce the dependence of the K-means clustering algorithm on it. Then, based on the processing method of representative points, the ideal clustering results can be obtained by selecting the global optimal solution in the clustering results. It is necessary to improve the selection of the initial cluster center in the selection of the initial cluster center of the clustering algorithm.

### 4.4. Problems Existing in the Introduction of New Products of Semiconductor Companies

As the primary consideration of the new product introduction work of semiconductor enterprises, the plan is an effective guarantee for the smooth progress of the new product introduction project and can guarantee the improvement of the business efficiency and management efficiency of the enterprise to a large extent. In the process of import management of new products, the development process, import process, and import of process modules of new products need detailed plans as support to realize the import of new products in the overall planning and scheming and to determine the relevant budget standards for manpower, material resources, and financial resources required for each work task and link.

The core of the new product introduction work of semiconductor companies is also mainly determined by the master plan of product introduction, which is not only constrained by the new product development process plan but also provides a basis for making plans for each functional module of the new product introduction. The new product introduction master plan is the baseline of the new product introduction management, and it is the basis for the control of the new product introduction progress, plan deviation, and preventive management. However, in the process of introducing new product F, there is a lack of corresponding plan management connection between the main plan and the import plan of each functional module in semiconductor companies, which leads to the problem of insufficient plan integration between different levels, specifically reflected in the following aspects:

First of all, as the core organization of new product introduction management, the production planning room of semiconductor companies did not clarify the corresponding relationship between the new product introduction master plan and each level plan in the early stage of new product introduction but was included in the unified management scope, and there is a lack of specific plan executives who are actively pulling, resulting in one-sidedness and lag between plan formulation and actual update. Secondly, the current plan management process of semiconductor companies is not standard enough for the review cycle of plans, and it is impossible to realize real-time monitoring and change analysis of new product introduction activities, which in turn affects the determination of evaluation results and the adoption of adjustment measures, which is not conducive to the coordination and unity of work objectives, tasks, and time, and it is not conducive to the stable progress of the new product F introduction management work and even delays the work progress.

## 5. Conclusions

With the vigorous development of semiconductor integrated circuits in recent decades, major international giant chip manufacturers have accelerated the research and development of the latest technology. Countless undercurrents and risks come with the opportunity. In this case, the analysis of systemic risks in the international semiconductor market becomes crucial. This paper deeply thought about the shortcomings of the original risk evaluation system starting from such a practical problem and proposed the topic of using the K-means algorithm based on deep feature fusion to analyze the systemic risk of the semiconductor global market. In the aspect of system optimization, the article carried out the data set retrieval results, used the correlation analysis function in R software to carry out correlation analysis on the selected data variables, and carried out K-means clustering center, K-means weighted clustering center, and a table of cluster center points. The experimental results showed that the average size of Category 3, Category 4, Category 6, and Category 7 was small, of which Category 7 had a faster growth rate, Category 3 and Category 6 were relatively stable, and Category 4 was shrinking in size; the average size of Category 1, Category 2, Category 5, and Category 9 was medium, of which Category 1 had a faster growth rate, Category 2 and Category 5 fluctuated slightly, and Category 9 was relatively stable; Category 8 had the largest average size and was the leading company in the semiconductor industry. The results are consistent with the facts, and the work has been completed well. In future experiments, it can be tried to add the implementation of risk estimation to the system and numerically represent the risk probability, which makes the system more visual and interactive.

## Figures and Tables

**Figure 1:** The SWOT matrix.

**Figure 2:** Thedynamic risk identification algorithm based on deep feature fusion characteristics.

**Figure 3:** Cluster fusion.

**Figure 4:** Semiconductor manufacturing process.

**Figure 5:** Basic statistics of yield.

**Figure 6:** ACF and PACF coefficients for yield series.

**Figure 7:** Comparison of stock risks of two semiconductor companies.

**Figure 8:** Number of clusters.

**Figure 9:** Number of clusters after weighting.

**Table 1:** Dataset retrieval results.

Characteristic dimension	VLAD	Fisher vector	Neural codes	MOP-CNN	OR-fused	Object feature pooling	Proposed
32	48.4	48.6	68.3	—	—	74.0	**76.6**
64	52.3	52.0	72.9	-	—	80.7	**81.4**
128	55.7	56.5	78.9	—	—	85.1	**87.5**
256	—	—	74.9	—	—	87.8	**91.4**
512	59.8	61.0	74.9	—	82.8	88.5	**92.0**
1024	—	—	—	—	83.7	86.6	**89.0**
2048	62.1	62.6	-	80.2	83.7	85.9	**89.7**
4096	55.6	59.5	79.3	78.9	—	85.9	**89.7**

**Table 2:** Thecorrelation coefficient table.

	Size	Compound growth rate	Coefficient	Active rate	MDU	Number of starts	Time	Time variation coefficient	Retention	Conversion rate	Unloading conversion
Average size	1.00										
Compound growth rate	0.04	1.00									
Coefficient of variation	−0.08	−0.29	1.00								
Active rate	−0.09	−0.12	0.46	1.00							
MDU	0.93	0.06	−0.12	−0.11	1.00						
Number of starts	0.98	0.03	−0.06	−0.07	−0.06	1.00					
Time	−0.08	−0.14	0.89	0.43	1.00	-0.06	1.00				
Time variation coefficient	0.98	0.03	−0.07	−0.07	−0.05	0.89	−0.06	1.00			
Retention	−0.08	−0.16	0.87	0.46	0.11	−0.26	0.11	−0.28	1.00		
Conversion rate	0.13	0.22	−0.32	−0.47	0.17	0.11	−0.26	0.11	−0.28	1.00	
Unloading conversion	0.00	0.06	−0.03	−0.01	−0.01	0.00	0.01	0.00	0.00	0.13	1.00

**Table 3:** K-means cluster centers.

Category	Number of clusters	Average size	Compound growth rate	Coefficient of variation	Active rate coefficient	Retention	New installation conversion
Category1	316	−0.06	0.29	−0.64	−0.44	−0.43	0.24
Category2	337	0.12	0.41	−0.87	−0.83	1.13	0.25
Category3	184	−0.08	−0.77	0.38	−0.10	−0.73	0.33
Category4	186	−0.06	−0.21	−0.12	−0.39	−0.28	−1.82
Category5	104	−0.08	1.10	0.54	1.44	−1.08	−0.29
Category6	2	26.85	0.50	−1.41	−1.61	2.10	-0.06
Category7	74	−0.05	2.22	0.99	−0.20	0.65	0.20
Category8	124	−0.07	0.27	−0.30	0.76	0.66	0.58
Category9	139	−0.08	−0.76	0.58	1.78	−1.04	−0.03
Category10	101	−0.08	−1.61	2.31	0.72	−0.60	−0.15
Category11	125	−0.07	−0.73	0.38	−0.26	0.95	0.65

**Table 4:** K-means weighted cluster centers.

Category	Number of clusters	Average size	Compound growth rate	Coefficient of variation	Active rate coefficient	Retention	New installation conversion
Category1	122	−0.11	2.03	1.03	0.34	0.02	0.14
Category2	169	0.00	−0.20	−0.09	−0.42	−0.03	−1.96
Category3	326	−0.14	−0.61	0.32	0.02	0.48	0.81
Category4	152	−0.15	−1.47	1.92	0.96	−0.64	0.12
Category5	446	−0.03	0.35	−0.77	−0.56	0.06	0.10
Category6	27	−0.13	−0.50	−0.03	−0.09	−0.72	0.22
Category7	207	−−0.14	0.12	0.13	1.67	−0.88	−0.14
Category8	7	13.02	0.62	−1.20	−1.33	1.58	−0.59
Category9	236	0.22	0.39	−0.76	−0.87	1.68	0.37

**Table 5:** Cluster center points.

Category	Number of clusters	Average size	Compound growth rate	Coefficient of variation	Active rate coefficient	Retention	New installation conversion
Category1	122	−0.06	1.74	0.77	0.15	0.31	0.17
Category2	165	−0.01	0.07	−0.08	−0.36	0.05	−1.55
Category3	182	−0.14	−0.63	0.23	−0.02	0.04	0.73
Category4	153	−0.15	−1.53	1.99	0.88	−0.56	0.12
Category5	419	−0.01	0.30	−0.76	−0.57	0.04	0.07
Category6	259	−0.11	−0.56	0.21	0.16	−0.62	−0.45
Category7	190	−0.14	0.14	0.11	1.61	−0.87	−0.10
Category8	7	13.02	0.62	−1.20	−1.33	1.58	−0.59
Category9	195	0.09	0.70	−0.31	−0.57	1.33	0.31

## Data Availability

This article does not cover data research. No data were used to support this study.
